RETRACTED

# The Dynamic Movement of Disaster Management Systems Based on Vehicle Networks and Applied on the Healthcare System

**DOI:** 10.1155/2021/5710294

**Published:** 2021-10-16

**Authors:** Malik Bader Alazzam, Fawaz Alassery

**Affiliations:** ^1^Faculty of Computer Science and Informatics, Amman Arab University, Jordan; ^2^Department of Computer Engineering, College of Computers and Information Technology, Taif University, Taif, Saudi Arabia

## Abstract

In order to save human life and assets, the emergency management system (DMS) requires roving rescue teams to respond promptly and effectively. Installation and restoration of appropriate communication infrastructure are important for reducing the effect of disasters and enabling and coordinating information flow among relief teams working in the region. This paper describes a data collection system based on vehicular cloud network services that incorporates the advantages of both architectures of vehicular ad hoc networks (VANETs) with the cloud to establish vehicular cloud networks (VCNs). Vehicles in the current plan perform tasks like monitoring the environment, gathering data, and transmitting data to the control center depending on their positions and instructions. To build a disaster management system, the proposed system uses hybrid wireless networking, which includes both a central system and ad hoc networks. The implementation results show that the suggested system is more dependable and efficient; even light density is improved in terms of reachability with few hops. Furthermore, as compared to the existing system, the suggested system has a lower end-to-end delay and a higher packet delivery ratio.

## 1. Introduction

Every year, the globe faces a major challenge when different catastrophic natural catastrophes, such as tsunamis, typhoons, hurricanes, and earthquakes, strike. Natural disasters have fully or partially devastated certain areas, making them hazardous for human life. Great financial and human losses were recorded in these situations, as well as the impact on every one of these needed to be minimized (economic, human). The cost of the recent earthquake and tsunami in Japan is projected to be over $300 billion USD [1]. Many countries, however, have begun to implement a system that addresses these issues. Individuals and authorities, of one, must engage with each other under such conditions for a number of reasons, ranging from seeking a safe sanctuary to discovering secure routes. Rescue and other efforts have been delayed and impeded as a result of the communication system's collapse. Furthermore, because of the breakdown in communication, there is a lack of communication between people, authorities, and organizations and disaster relief personnel [2].

RETRACTED

As a cornerstone of the connecting system to ease rescue operations, communication structure is considered. The most important duty for this kind of networks is to gather critical information in order to locate and rescue people. The probable survivors' location, as well as the intended subjected to retrieve the trapped individuals in every place, is analyzed in order to efficiently supply resources. Both of them are critical problems in any rescue operation. Maintaining network connectivity in order to collect relevant information and determining the location is not assured during or after a disaster. Worst of all, network connectivity is uncertain owing to the disaster's unanticipated infrastructure devastation. As a result, it is critical to look for a communication system that still works in such locations. We recognized the following concerns [3] that drive our research based on our observations. The solution needs to deploy and cover all the emergency zones without human intervention.

The new solution should be easy and uncostly to develop, and it should work for at least 72 hours until other communication network services are installed or restored. It is hard to use the Internet access for disaster rescue network and we can mitigate the dependable on connectivity by seeking for other resources.

We envision a large-scale disaster scenario in which existing terrestrial communication infrastructure is entirely destroyed. Many academics have offered numerous ways to solve this issue in the literature, but they all presume that a telecommunications operator is an integral element of their emergency management systems. We propose that a vehicular ad hoc network (VANET) can help bridge this gap. When VANETs and cloud computing are coupled, a vehicular cloud network (VCN) is formed, which allows cars to connect and share resources via a cloud platform. VCN applications have sparked a lot of interest in the previous ten years, especially when a new advanced technology has backed them up [4]. These facilities begin with safety and then go on to fascinating, cost-effective, and other features. One of these new emergency technologies is the smart car, which is packed with a lot of computing, storage, and processing power. These vehicles will increasingly be employed in a variety of applications that need VCN. In our suggested approach, however, a smart car is regarded as a mobile cloud server [4].  Figure 1 illustrates our perspective on the proposed disaster management system. DMS is set up with VCN, which includes cellular and ad hoc wireless networks. Inside each zone, cellular mode is used to gather data, while ad hoc mode is used to send data to the operations center (authority management).

RETRACTED

## 2. Previous Study

One of the most essential issues in an emergency situation is gathering essential information in a safe and timely manner in order to minimize damage and save the victims. The primary goal of data collecting systems is to prevent undue damage to critical lifeline infrastructure. Lifeline facilities such as mobile carriers, water supply, and electricity supply are examples of critical infrastructure that must be protected in such scenarios. Unfortunately, severe disasters throughout the world have repeatedly revealed flaws in data collecting systems that should allow for dependable communication among rescuers (emergency teams and relief agencies). In this field, several researches have been conducted.

With the help of other writers, Barik et al. [5] presented the SAFIRE system, which addressed the accessibility and flexibility of data transmission in emergency situations. SAFIRE uses a new multihop architecture to let first responders exchange information more quickly and reliably. SAFIRE's main characteristics include a decentralized platform, publish-subscribe data sharing, and multilayer designs that are adaptable. The major goal of this article is to achieve interoperability across multiple communication systems; however, there is no assurance that such systems will continue to operate in such an environment, which is a disadvantage.

Some writers emphasized pre- and postdisaster breadth conditions. Tripathi [6] proposed the RescueME system, which is linked with other current infrastructure communication networks to give a manner and entities for users to record their whereabouts. Many responsibilities and tasks are assigned to entities during a catastrophic event. For example, when natural disasters strike, the suggested system considers users to be drivers, but when disasters occur, users become potential survivors. The suggested solution to secure location data using public key infrastructure involves privacy and security. This research does not highlight or address communication system outages that occur as a result of disasters.

Zhang et al. [7] suggested the DistressNet system, which focuses on the needs of search-and-rescue professionals in the event of a crisis in an urban setting. Various devices, such as smartphones and low-power sensors, were combined into an easy-to-deploy infrastructure by the system. The total efficiency of the suggested system might be improved by the simple placement of these devices at specific optimum places near to the catastrophic region. Despite the authors' independent evaluations of numerous system components, the TestBed was performed without a full implementation. In addition, the DistressNet system employed an IEEE802.11a/b/g/n backbone networking stack with an Autonomous Basic Service Set (IBSS) phase. Furthermore, the system made use of a number of hardware motes, although IEEE 802.11 does not support them, such as Explicitly Parallel Instruction Computing (EPIC).

RETRACTED

Another research was conducted. Hameed et al. [8] built an Integrated Emergency Information Exchange (IECM) for catastrophe areas by combining wireless sensor networks with mobile ad hoc networks (MANETs). Based on the Integrated Emergency Service System, the proposed system delivers different emergency management services for rescue team members (IESS). Wireless mash networks IEEE 802.11s were used to configure mesh access points and mesh clients for MANETs. The end user chooses a connection path through MANETs, cellular networks, or satellite networks, if available, based on service requirements and network circumstances. In this case, it appears that this technique is unworkable in practice.

To discover the best evacuation tactics, Hamad et al. [9] presented an intelligent evacuation system. The major goal is to improve vehicular DMS by updating the transport management reaction. The authors concentrated on the suggested technique for evaluation, which is anticipated in dynamic decision-making in terms of efficacy evacuation features. However, this study does not address communication under a worst-case scenario in which communication services have failed, which is considered a cornerstone of any DMS.

In [10], Khalaf et al. develop an intelligent traffic-related cloud disaster management system (IVCDM) concept that supports multimode communication to keep cars connected. V-I (vehicle-to-infrastructure), V-P (vehicle-to-pedestrian), and V-V (vehicle-to-vehicle) are three multimode communication approaches for message transmission. To assess the proposed system city and highway environment, two scenarios are considered. The findings show that connection in the V-P mode is more efficient than that in the V-V mode. Actually, the article does not address city-environment connection. In this V-P mode, the paper assumes that communication systems continue to function in catastrophe scenarios when connection is not assured.

Finally, Khader and Eleyan [11] created an emergency plan for a TestBed implementation that relied on VANET connections. The authors focus on communication among rescue teams in situations where no system can be utilized for communication. TestBed is an application that is used to communicate important information via VANET environments for this purpose. TestBed is equipped with onboard devices that include a credit card-sized microprocessor called the Raspberry Pi, as well as a Global Positioning System, to allow cars to engage in the proposal system. Furthermore, messages were sent across many hops on their route to the central control unit using predefined code based on the amount of urgency. As a result, the authority takes proper action based on the message code received from the client. The system was evaluated based on a variety of criteria, including network latency and dependability in relation to the number of hops, and its applicability was demonstrated. Finally, the system makes no mention of the vehicle arrangement inside the scenario or interest area.

RETRACTED

In all of the above cases, a working or a standby communication system in place can highly reduce the impact of catastrophic situation.

Challenges and system requirements: the major system requirements and challenges that need to take an account to establish network connections for sharing information for disaster rescue system are listed below.

Intermittent connectivity: the damages in the infrastructure are unforeseeable and the connectivity is not predictable. The delivery of the information is not reliable and not guaranteed. The intermittent faculty in connectivity or communication may occur partially or totally; sometimes the region is isolated [2]. In such situation, more reasonable turn form end-to-end delivery to continual storage and redundancy storage. This approach of storing requires saving the sharing information in available resources so that it will later reach the rescue network. Redundancy storage requires storing the information in a distribution fashion.

Consuming idle vehicle resources in VANET platform is the basic idea behind the concept of VCN. Vehicle resources are leveraged, and the capabilities of the vehicles like sensing, data storage, relaying information, computing, and other facilities allow the vehicle to perform as mobile service provider. With these added new components, a vehicle represents as an intelligent vehicle which supports many services. The authors in [2, 11–18] introduce vehicle as a resource (VaaR) which adopted various vehicular potential services. According [3, 4, 6, 19] to authors' point of view, the vehicle can provide various instances of VaaR.

## 3. The New System

When an unforeseen disaster strikes a specific location, several assumptions must be made in order to design a system to deal with the situation. One of the most important assumptions is that the city region would be divided into tiny zones that can be readily managed. Every zone is surrounded by a barrier line that separates it from its neighbors. A digital map that includes these zones is considered virtual mapping (digital map) that is stored implicitly from every smart (intelligent) car wandering the city. However, in the case of a crisis, these smart cars are dispersed at random around the city, with the assumption that the communication network will fail. As previously said, the best communication architecture is one that can stay operational for as long as feasible. When tragedy strikes, VANETs are the least affected platform in contrast to other communications networks. As a result, in a chaotic environment, the link between all smart cars is critical to keeping the communication system running as smoothly as possible. We choose three varieties of VaaR to perform in our suggested system this way: storage and computation of VaaR data (VaaR-Storage), relaying of VaaR data (VaaR-Relaying), and sensing of VaaR data (VaaR-Sensing). Each of them has a specific role to play in our system, which includes monitoring the zone environment, collecting monitoring data, and eventually forwarding data to neighboring zones via VaaR-Relaying nodes. The proposed system uses a varied VaaR, and the following is a detailed explanation of each of them.

RETRACTED

VaaR-Storage (data center): this sort of vehicle aggregates data within each zone. This kind functions as a data server, collecting data from nearby VaaR-Sensing cars. The center occupancy at every zone is imposed by the VaaR-Storage vehicle's mission. The amount of VaaR-Storage in each zone must include at least one that is chosen based on their location. VaaR-Storage then sent the data to the relaying node, which serves as an interface to other zones.

## 4. Model of a Network

Figure 2 illustrates the proposed vehicular cloud network layered approach. Each layer has specific task which is related to a type of vehicle cloud service provider. The components of each layer have distinct task and their locations so the role of them is different as well. The system suggested that the wireless communication technology dedicated shorted-range communications [2–4, 11, 18, 19] is a medium between any two layers with one-hop distance separating them.

As mentioned previously, the city is classified into various zones, and each zone involved a network of roads and intersections. All this information is stored in the digital map which is saved in all smart vehicles. The most significant coordinates are the center and boundary of zones. Through these coordinates, the smart vehicle will play the VaaR-Storage and VaaR-Relaying node role.

## 5. Preparation Phase

In this phase, in case the emergency occurs, all smart vehicles (VaaR) have a built-in virtual map of the city. According to proposed network model of the system, VaaR are randomly distributed in the city and assumed equipped with Global Positioning System [13]. Every VaaR can play different roles according to their location; VaaR close to the zone center play as a VaaR-Storage, while VaaR near the zone border play as a VaaR-Relaying node; between center and border zone, the VaaR-Sensing are disseminated randomly through the zone. To identify the location of each VaaR in the zone, the below strategy is used.

RETRACTED

Each vehicle will send a message to advertise their location to all one-hop neighbor. This message contains VaaR location and direction. Figure 2 depicts the content of the message. All vehicles issue a neighbor list and update it periodically and save it as a history of movement. Thus, VaaR can calculate its direction using

(1) $$\begin{array}{c} \beta =\tan^{-1}\frac{Y2-Y1}{X2-X1}, \end{array}$$

where (*X*2, *Y*2) is the current coordinate of the VaaR at *t*2 time, (*X*1, *Y*2) is the previous coordinates at time *t*1, and *β* is the VaaR heading angle which represents the direction of the VaaR. The information of message in this step is shown in Figure 2.

After this step is completed, each VaaR knows its location with respect to zone coordinates, and according to Algorithm 1, the VaaR plays either VaaR-Storage, VaaR-Relaying, or VaaR-Sensing. This phase involved cellular network formation mode when VaaR-Storage while VaaR-Relaying identification.

## 6. Phase of an Emergency

When each member of the zone is recognized: VaaR-Storage, VaaR-Relaying, and VaaR-Sensing, the second phase begins. Reading the environment zone and flow information from VaaR-Sensing vehicle is starting. VaaR-Storage accepts the data from all zone members' vicinity to aggregate and collect them. Furthermore, VaaR-Storage is ready to forward data to VaaR-Relaying node which in turn forwards the data to other VaaR-Relaying node in other zones in the way to authority manager. In this way, the ad hoc wireless network mode is established by distinguishing the available route to authority management. The routing protocol IAODV is in [6]. Here, studs were showing or are used to deal with looking for route from VaaR-Relaying to another and finally to authority management. The content of emergency message are zone ID, first delayered ID, second relayed ID, emergency data, number of hops, and timestamp as shown in Figure 2 Whether VaaR-Relaying is the first delayered or the second one depends upon the format field of emergency message. In case of message relaying twice, the format field of emergency message assures the second relaying ID and so on. Each delayered node adds its ID and increases the hop count by one.

RETRACTED

## 7. Result Analysis

Figure 3 depicts the relationship between reachability and the number of hops tallied in order to evaluate the suggested system. The rate at which data from VaaR-Sensor nodes reaches management authorities is referred to as reachability. As a result, the influence of the number of hops has a noticeable impact on the system's behavior. Reachability diminishes as the number of hops rises, due to multihopping, which causes link breakage. Due to degradation or disturbance of the propagation model, these connections are susceptible for a variety of reasons. In addition, as the number of hops rises, the link relationship may deteriorate. As a result, when excessive hops are needed in link creation, the network's dependability suffers.

Figure 1 depicts three distinct densities: low, midrange, and high density, with their influence on reachability clearly highlighted. When density is large, reachability increases to 100%, especially for VaaR-Sensor networks that are close to management authority (one hop count). For other nodes where multihopping is required to reach authority administration reachability levels, another ratio degradation occurs.

Furthermore, two metrics for performance assessment of the two situations with vehicular cloud (with VC) even without automobile cloud (without VC) are chosen (without VC). The first was about the sender node with receiver authority management's end-to-end (E-2-E) message delay time. The packet delivery ratio (PDR) between source and destination is the second statistic. Both the E-2-E delay and the PDR are critical measures for demonstrating efficiency in an emergency circumstance. The suggested system's major aim is to rapidly and reliably send emergency information about the environment to authority management. As a result, these measures were chosen to represent performance and resilience to difficult conditions when data transfer must be managed and handled carefully.

The relationship between PDR and simulation time is seen in Figure 4. PDR refers to the amount of packets that arrive at the authority management in relation to all transmitted packets. The proposed method (with VC) achieves good performance with only 5 hops, whereas the existing approach (without VC) requires 10 hops or less, resulting in PDR deterioration. The reason for this is that existing systems require a multihop link, but the suggested method does not.

Where the humanistic lives are at risk, real-time links are critical in rescue networks.  Figure 5 delays in transportation environment information result in a large number of individuals becoming lost.  Figure 2 depicts the differences in behavior between the proposed and existing systems when transmitting emergency data. The suggested system has a lower average E-2-E latency than the traditional system. As previously stated, linkages with numerous hops take longer and are more prone to distortion, whereas connections with few hops do not. This study suggested a web analytics system for disasters that is based mostly on the VANET architecture.

RETRACTED

## 8. Conclusion

This study suggested a web analytics system for disasters that is based mostly on the VANET architecture, where member nodes are distributed at random around the city and participate in the formation of a rescue network. The suggested system is based on hybrid wireless connectivity and includes a cellular network and an ad hoc network. Cellular networking is utilized within the zone, while ad hoc wireless connections are used between relay nodes (gateway) on the route to authority management. The suggested system is thought to cover the emergency situation reporting environment using this technique. Simulations show that the suggested system's reachability is more efficient than a standard system with a lower hop count. The suggested system can provide great reachability with only 5 hops, whereas typical systems require at least 10 hops to obtain the same reachability. Traditional systems do not provide considerable reachability at varying densities, but the proposed approach does. Furthermore, in the case of average E-2-E latency and PDR metrics, the suggested system performs flawlessly to meet the primary goal of establishing a rescue network.

Future work will be necessary to improve the suggested system in many ways. The position of the relay vehicle is critical for routing data to the operation center, and this element must be thoroughly investigated. Another consideration is the amount of time VaaR-Storage and VaaR-Relaying must wait to complete their tasks, which necessitates thorough research.

## Figures and Tables

**Figure 1:** Outline of the disaster management system.

**Figure 2:** The proposed network model.

**Figure 3:** Reachability versus no. of hops.

**Figure 4:** PDR versus simulation time.

**Figure 5:** E-2-E delay versus simulation time.

**Algorithm 1:** Selecting VaaR-Storage and VaaR-Relaying vehicles.

## Data Availability

The data underlying the results presented in the study are available within the manuscript.
